The article "Randomised controlled trial of a home-based physical activity intervention in breast cancer survivors" was published in 2016. Journal: BMC Cancer.

# Randomised controlled trial of a home-based physical activity intervention in breast cancer survivors

**DOI:** 10.1186/s12885-016-2258-5

**Published:** 2016-03-17

**Authors:** Ian M. Lahart, George S. Metsios, Alan M. Nevill, George D. Kitas, Amtul R. Carmichael

**Affiliations:** Faculty of Education, Health and Wellbeing, University of Wolverhampton, Walsall Campus, Gorway Road, Walsall, WS1 3BD UK; Department of Surgery, Russells Hall Hospital, Dudley, DY1 2HQ UK; Department of Research and Development, Dudley Group NHS Foundation Trust, Russells Hall Hospital, Dudley, DY1 2HQ West Midlands UK

**Keywords:** Breast neoplasms, Physical activity, Randomised controlled trial

## Abstract

**Background:**

To improve adherence to physical activity (PA), behavioural support in the form of behavioural change counselling may be necessary. However, limited evidence of the effectiveness of home-based PA combined with counselling in breast cancer patients exists. The aim of this current randomised controlled trial with a parallel group design was to evaluate the effectiveness of a home-based PA intervention on PA levels, anthropometric measures, health-related quality of life (HRQoL), and blood biomarkers in breast cancer survivors.

**Methods:**

Eighty post-adjuvant therapy invasive breast cancer patients (age = 53.6 ± 9.4 years; height = 161.2 ± 6.8 cm; mass = 68.7 ± 10.5 kg) were randomly allocated to a 6-month home-based PA intervention or usual care. The intervention group received face-to-face and telephone PA counselling aimed at encouraging the achievement of current recommended PA guidelines. All patients were evaluated for our primary outcome, PA (International PA Questionnaire) and secondary outcomes, mass, BMI, body fat %, HRQoL (Functional assessment of Cancer Therapy-Breast), insulin resistance, triglycerides (TG) and total (TC), high-density lipoprotein (HDL-C) and low-density lipoprotein (LDL-C) cholesterol were assessed at baseline and at 6-months.

**Results:**

On the basis of linear mixed-model analyses adjusted for baseline values performed on 40 patients in each group, total, leisure and vigorous PA significantly increased from baseline to post-intervention in the intervention compared to usual care (between-group differences, 578.5 MET-min∙wk^−1^, *p* = .024, 382.2 MET-min∙wk^−1^, *p* = .010, and 264.1 MET-min∙wk^−1^, *p* = .007, respectively). Both body mass and BMI decreased significantly in the intervention compared to usual care (between-group differences, −1.6 kg, *p* = .040, and −.6 kg/m^2^, *p* = .020, respectively). Of the HRQoL variables, FACT-Breast, Trial Outcome Index, functional wellbeing, and breast cancer subscale improved significantly in the PA group compared to the usual care group (between-group differences, 5.1, *p =* .024; 5.6, *p* = .001; 1.9 *p* = .025; and 2.8, *p =* .007, respectively). Finally, TC and LDL-C was significantly reduced in the PA group compared to the usual care group (between-group differences, −.38 mmol∙L^−1^, *p =* .001; and −.3 mmol∙L^−1^, *p =* .023, respectively).

**Conclusions:**

We found that home-based PA resulted in significant albeit small to moderate improvements in self-reported PA, mass, BMI, breast cancer specific HRQoL, and TC and LDL-C compared with usual care.

**ClinicalTrials.gov identifier:**

NCT02408107 (March 25, 2015)

## Background

Worldwide, breast cancer is the most frequently diagnosed cancer and the leading cause of cancer death among females [1]. In the UK, female breast cancer has the highest incidence rate of all cancers [2], and is predicted to increase by 44 % up to 2020 [3]. Owing largely to early detection and improved treatment strategies, UK breast cancer mortality rates are falling [4], resulting in the largest prevalence of breast cancer survivors in the UK ever reported.

Due to the prevalence of treatment-related health concerns and increased risk of developing metabolic syndrome, recurrence and cardiovascular disease, breast cancer survivors may require diagnostic, therapeutic, supportive or palliative services for many years post-diagnosis [5–7]. Encouraging breast cancer survivors to adopt a healthy lifestyle post-treatment may reduce the healthcare burden resulting from treatment-related sequelae and improve survival [8]. In particular, higher levels of physical activity (PA) may reduce risk of recurrence and all-cause and breast cancer-related mortality [9–12]. However, PA levels are generally low among breast cancer survivors and many women decrease their PA following diagnosis [13–15]. Therefore, interventions are required to improve the post-diagnosis PA levels of breast cancer survivors.

Randomised controlled trials (RCTs) have found improvements in PA levels, cardiorespiratory fitness, HRQoL, fatigue and weight maintenance in breast cancer survivors participating in PA interventions compared with control groups [16–27]. However, most PA RCTs consist of either entirely or partly facility-based interventions, and therefore, the findings of these trials may not generalise to patients who have limited access to exercise facilities because of transportation, time-related and financial difficulties [22]. In addition, facility-based studies may lack external validity, or real world application, which limits the translation of their findings into practice [28]. To overcome this problem some trials have provided entirely home-based PA interventions [17, 18, 20, 22, 24–27]. In addition to mitigating transport, time-related and financial difficulties, home-based interventions are also advantageous because they are less expensive than supervised, facility-based interventions and do not require participants to attend classes or maintain a health club membership to sustain PA [22].

For breast cancer survivors to maintain their PA participation during and after the specified intervention period, it is important that they are given behavioural change support [19]. However, only three home-based intervention trials included a specific PA behavioural change support component, consisting of both face-to-face counselling and support telephone calls [17, 20, 27]. Although the findings of these home-based PA trials are promising, they had a number of limitations (small sample sizes and short intervention duration of 12 weeks, [17, 20, 27]; postmenopausal women only, [17, 27]) that limit the generalizability of their results. Therefore, the aim of this current study was to investigate the effects of a pragmatic (i.e. designed to test the effectiveness of an intervention in a broad routine clinical practice, [29]) 6-month home-based PA intervention with counselling on PA levels, weight maintenance, HRQoL, and blood biomarkers in breast cancer survivors.

## Methods

### Participants

Women attending breast cancer clinics between January 2010 and March 2013 at Russells Hall Hospital (Dudley Group NHS Foundation Trust, UK), were invited to participate. Participants were eligible to participate if they were: 1) females aged 18–72 years, 2) diagnosed with invasive breast cancer (Stage I–III) within two years of enrolment, 3) post-surgery and had no surgery planned for the next six months at least, 4) had fully completed adjuvant therapy (radiotherapy and/or chemotherapy) not including hormonal therapy, 5) no previous malignancy, 6) willing to be randomised 7) and willing to maintain contact with the investigators over the six months. Exclusion criteria included: 1) inability to participate in PA because of severe disability (e.g. severe arthritic conditions), 2) psychiatric illness and 3) vulnerable subjects, such as pregnant women or any other patient where PA was not approved by their oncologist due to the presence of one or more contraindications to exercise in cancer patients [30]. Participants who were physically active at the time of enrolment were not excluded from participation. The study was approved by the Black Country NHS Ethics Committee. All participants provided written consent prior to data collection.

### Randomisation

At a Clinic Trials Unit on a different site, a computer generated random numbers list was used to allocate all participants into intervention or usual care groups (concealed from the primary researcher), and allocate 40 % of participants in each group into a substudy involving cardiorespiratory fitness assessment (data not reported). Patients were allocated to intervention and usual care groups on a 1:1 ratio and were stratified based on adjuvant chemotherapy. Randomisation occurred after participants had completed baseline questionnaires and had a blood sample taken.

### Home-based PA intervention

Following randomisation, patients received an intervention aimed at encouraging the adoption of a more physically active lifestyle. Participants received a face-to-face consultation, followed by a support telephone call at the end of months one, two and three (i.e. a total of 3 telephone calls). During each of the last two months (4 and 5) patients received a mailed PA reminder leaflets encouraging their participation in home-based physical activity. The intervention was based on the findings from previous research [31, 32], which suggested that breast cancer survivors had strong preferences for the receipt of face-to-face counselling from exercise professionals and for moderate-intensity PA at home and/or outdoors.

Face-to-face consultations were conducted by the primary researcher immediately after initial baseline measurements and were based on the four core motivational interviewing principles: expressing empathy, developing discrepancy, rolling with resistance and supporting self-efficacy [33, 34]. To ensure consistency in intervention delivery, a semi-structured motivational interviewing-based intervention protocol was developed to guide intervention delivery. The topics covered in the 30–45 min consultation were similar to other trials that incorporated a PA counselling component [17, 20, 22, 27], including: current PA behaviour, decision balance exercise; benefits of PA in general and specific to breast cancer survivors; perceived barriers; prompts to seek social support, goal setting, types and intensities of PA (e.g. explanation of light, moderate and vigorous PA with examples specific to participants, such as, taking a brisk walk so that you are mildly breathless but can still hold a conversation); safety advice; and basic lifestyle information (e.g. basic dietary information, portion size, fat intake, smoking, and hydration in generally and during activity).

The focus of the follow-up phone calls (end of months 1–3) was to prevent relapse back to inactivity and/or improve maintenance of PA (accumulate 30 min of moderate-intensity PA on 3–5 days/week), and covered topics similar to the face-to-face consultation. Calls lasted approximately 15–20 min and were guided by standardised phone call scripts. Participants were encouraged to telephone the research team should they encounter any problems or relapse in their efforts to increase their PA. Therefore, our intervention represented a pragmatic step down approach (i.e. from in-person sessions to telephone calls to postcard prompts), that could feasibly be employed by cancer care nurses in routine clinical practice.

The initial goal of the intervention (months 1–3) was for participants to progress towards accumulating 30 min of moderate intensity PA on three to five days per week. During months three to six, the intervention participants were encouraged to work towards accumulating at least 30 min of moderate-intensity PA on five to seven days per week in broad agreement with current public health guidelines [35]. If participants were already achieving this on trial entry they were, as a minimum, actively encouraged to maintain their level of PA. Participants were encouraged to first focus on the frequency of their PA and then duration.

Participants were given a PA pack consisting of an information booklet and a DVD (previously developed by Breast Cancer Care) that provided further information of topics such as exercising safety, exercise intensity, dealing with fatigue and exercising with lymphedema. Information about local physical activity opportunities was also provided, including an exercise initiative run in local parks. During the intervention period, participants were encouraged, but not required to keep PA diaries to check against whether they were achieving 150 min of moderate-vigorous PA over each week. Participants were advised to refrain from activity if they experienced any problems relating to the PA intervention (e.g. chest pain or developed a joint problem). If these circumstances occurred, patients would have been advised to contact the clinical team, and the clinician of the research team would have made a clinical decision based on the contraindications and precautions to PA for patients with cancer as to whether the patient refrained from PA temporarily or withdrew from the intervention [30].

### Usual care group

Participants randomised to the usual care arm received standard information regarding PA (i.e. current recommended PA guidelines), as provided to all breast cancer patients treated at the site. Usual care group participants were instructed to maintain their current lifestyle. After completion of the intervention participants in the usual care group were encouraged to adopt a more physically active lifestyle and were given the same guidance and physical activity pack as the intervention group.

### Outcomes

After randomisation, all participants’ had their height, mass and body composition measured and completed a demographics questionnaire, interview-administered long form International PA Questionnaire (IPAQ), Functional Assessment of Cancer Therapy-Breast (FACT-B) questionnaire and blood collection. The primary outcome of the current study was total PA (MET-min∙wk^−1^). Body composition (body fat %) was assessed after a 12-h water-only fast by bioelectrical impedance analysis (BIA) using a Tanita BC-418 MA Segmental Body Composition Analyser, which incorporates eight tactile electrode (Tanita Corporation, Tokyo, Japan). The specific device has a standard error of <3 % when standard procedures are followed [36]. Body mass was also measured via the Tanita analyser and was recorded to the nearest .1 kg. BMI (kg/m^2^) was calculated on the basis of measured height and mass. Standing height was measured without shoes to the nearest .5 cm on a portable stadiometer (Seca 214 Road Rod, Seca gmbh & co. kg., Hamburg, Germany).

Participants completed the validated IPAQ-long form questionnaire, which assesses the duration (number of days × hours/min per day) that an individual has engaged in walking, moderate, and vigorous PA across four domains (occupational, active transportation, domestic, and leisure) over the past seven days [37]. PA data were then used to calculate the metabolic equivalent (MET)-based IPAQ score by weighting each type of activity by its MET energy requirement (3.3 × walking duration; 4 × moderate PA duration; 8 × vigorous PA duration). Data were summed across activity domains to produce a weighted estimate of total PA (primary outcome) from all reported activities per week (MET-min∙wk^−1^), as well as subtotal of activity for each of the four domains, as well as walking, moderate and vigorous PA. The IPAQ allows individuals to be categorised into those who are meeting the current recommended PA guidelines (high and moderate PA categories) and those who are not (low PA category) [35]. Categorisation is based on the following algorithm: 1) high: vigorous PA on ≥3 days and accumulating ≥1500 MET-min∙wk^−1^, or ≥7 days of any PA accumulating ≥3000 MET-min∙wk^−1^; 2) moderate: vigorous PA on ≥3 days for ≥20 min/day, or moderate PA/walking on ≥5 days for ≥30 min/day, or ≥5 days of any combination of PA accumulating ≥600 MET-min∙wk^−1^; and 3) low: any combination of PA accumulating <600 MET-min∙wk^−1^. The IPAQ has good reliability (Spearman’s rho = .8) and moderate concurrent validity (Spearman’s rho = 0.33) when compared to accelerometer data (Spearman’s rho = .33) [37].

FACT-B is a 36-item compilation of questions subdivided into four primary HRQoL domains, including physical well-being (PWB; 7-items), social/family well-being (SWB; 7-items), emotional wellbeing (EWB; 6-items) and functional well-being (FWB; 7-items), and a disease specific domain, the breast cancer subscale (BCS; 9-items) [38]. The four primary HRQoL domains are combined to provide a 27-item general HRQoL assessment (FACT-G). The total FACT-B score is calculated by the sum of FACT-G and breast cancer subscale scores. The Trial Outcome Index (TOI), which provides an efficient summary index of physical/functional outcomes was also calculated as the sum of the PWB, FWB and breast cancer subscale scores. Possible score ranges were 0–36 for the BCS, 0–104 for the FACT-G, 0–140 for the FACT-B, and 0–92 for the TOI. Higher scores represent better quality of life or less severe symptoms. FACT-B has been validated in the breast cancer setting, with good internal consistency (alpha coefficient = .9), reliability, patient acceptability and sensitivity to clinically significant change [38]. All assessments were made at baseline and within two weeks of completing the 6-month intervention.

### Blood collection and laboratory analysis

Participants were instructed not to exercise for at least 28-h before blood collection. Blood was collected between 9:00 a.m. and 11:00 a.m. on the same day as other assessments after 12-h water-only fast. The Vitros® 5, IFS chemistry system (Ortho Clinical Diagnostics Inc., Rochester, New York, USA) was used to measure all lipid components; however, total cholesterol (TC), high-density lipoprotein (HDL-C), and triglycerides (TG) were measured using multi-layered slides, whereas measurement of low-density lipoprotein (LDL-C) required a dual chamber package. Plasma glucose was measured using the VITROS® 5.1 FS chemistry system (Johnson and Johnson Inc., Langhorne, PA, USA) and the same procedure as with cholesterol (but not LDL-C) was followed. Insulin was estimated from serum stored at −20 °C. The method of detection is a solid phase two-site chemi-luminescence immunometric assay. The Immunolite 2000 insulin was used on the Immulite 2000 Analyser (Siemens Healthcare Diagnostics, Deerfield, IL, USA). Homeostasis Model Assessment (HOMA) of insulin resistance (IR) was evaluated from fasting glucose and insulin [39].

### Sample size calculation and statistical analysis

Power calculations were based on total PA as the primary outcome. Using a between-group mean (SD) change in self-reported PA of 16.5 (25.1) MET-h∙wk^−1^ found in a similar trial [20], we estimated that with at least 36 participants in each group (*N* = 72), the trial would have 80 % power at *p* < 0.05. To allow for 10 % attrition we aimed to recruit 80 participants (40 in each group). Continuous variables were expressed as mean ± *SD*, while categorical data were presented as number of participants and percentages.

We used linear mixed-model analysis to examine the differences in the PA intervention group compared with the usual care group in changes over time from baseline to 6-month follow-up for all continuous outcome measures. Each analysis was adjusted for the baseline value of the outcome to control for between group baseline imbalances. Other covariates, including age, BMI (for non-anthropometric analyses), time since diagnosis (weeks), and time since treatment completion (weeks), were adjusted for but did not influence estimates so were not included. For each analysis, to select the best model, −2 log likelihood (i.e., maximum likelihood ratio test/deviance test) was used. Compared to a model with first-order, auto-regressive covariance structure for the repeated component (time) and a diagonal error covariance structure for the random effect (group), a model with unstructured variance for the repeated component and a compound symmetry for the random effect provided the best model, in all analyses. We used the intention-to-treat principle. For participants with missing data at post-intervention or follow-up, we included all available data under the missing-at-random assumption of the mixed-model analysis.

We performed per-protocol analyses among participants who completed both baseline and post-intervention assessments using a contemporary magnitude-based inferences approach [40]. In this approach, mean effects of the PA intervention and their 90 % confidence limits were estimated with a spreadsheet [41] via the unequal-variances *t* statistic computed for change scores between baseline and post-intervention in the two groups and adjusted for baseline values of each outcome. Each participant’s change score was expressed as a percentage of baseline score via analysis of log-transformed values, to reduce bias arising from non-uniformity of error. For this approach, effect sizes were calculated by dividing the log-transformed mean differences between intervention and usual care groups divided by the pooled log-transformed baseline SD of outcomes. The spreadsheet also computed quantitative and qualitative chances that the true effects were beneficial/positive, trivial, and harmful/decrease when a value for the smallest meaningful change was entered. A Cohen unit of .2 was employed as the smallest meaningful change in outcomes. Where the chance of benefit and harm are both >5 %, the effect is deemed *unclear*. Qualitative descriptors were then assigned to the quantitative percentile scores as follows: 25–75 % *possible,* 75–95 % *likely,* and >99 % *most likely*.

Chi-square analysis was planned on IPAQ categorical data but was not possible because greater than 20 % of the expected counts were less than five and some of the expected frequencies were below one. Collapsing the moderate and low categories into one category did not remedy this. Therefore, the PA data were presented as frequencies in those who completed post-intervention assessments. The FACT-B, FACT-G, TOI, and BCS HRQoL variables were categorised based on whether participants experienced a minimum clinically important (based on performance status and pain anchors) increase from baseline to post-intervention [42]. Chi-square analysis was then performed to examine intervention and usual care groups for differences in the number of participants who experienced a minimum clinically important increase in these variables. In the intention to treat analysis, standardized effect sizes were calculated for all outcomes by dividing the adjusted between-group difference of the post-intervention means by the pooled baseline standard deviation. According to Cohen [43], effect sizes <.2 indicate ‘no/trivial difference’, effect sizes of .2 to .5 indicate ‘small differences’, effect sizes of .5 to <.8 indicate ‘moderate differences’, and effect sizes ≥.8 indicate ‘considerable differences’. The level of significance was set at *p* < .05.

## Results

### Flow of participants through the trial and recruitment

Eighty participants were recruited for this trial between January 2010 and March 2013. Flow of participants through the study is provided in Fig. 1, including number of recruited participants and reasons of dropping out.

**Fig. 1:** Flow of participants through the trial

### Participant characteristics at baseline

Table 1 provides the baseline characteristics overall and by group assignment. Baseline data were collected from 80 breast cancer survivors (age = 53.6 ± 9.4 y; height = 161 ± 6.8 cm; mass = 68.7 ± 10.5 kg). The baseline characteristics of participants in the intervention and usual care groups were overall similar in most demographic (Table 1), anthropometric characteristics (Tables 1 and 2) HRQoL and biomarkers (Table 3), with only a few dissimilarities (e.g. usual care group reported more co-morbidities). Those in the usual care group were more physically active compared with the intervention group at baseline (Table 2), which was due mainly to a greater amount of domestic PA. Regarding IPAQ PA categories (Table 1), at baseline 15 % (*n* = 6) more participants were categorised in the high activity category in the usual care group compared with the intervention group. No adverse events were reported during the 6-month intervention period, although one participant in the usual care group dropped out due to PA unrelated-sciatica (see Fig. 1).

**Table 1:** Personal characteristics of the participants at baseline (intervention, *n* = 40; usual care, *n* = 40)

	Participants N (%) overall	Participants N (%) intervention	Participants N (%) usual care
Mean ± *s* age (y)	53.6 ± 9.4	52.4 ± 10.3	54.7 ± 8.3
Mean ± *s* time since diagnosis (weeks)	38.0 ± 20.8	42.2 ± 20.0	34.4 ± 21.1
Mean ± *s* weeks from end of treatment	10.5 ± 9.0	8.9 ± 7.3	12.0 ± 10.3
Ethnic origin:			
o White British	76 (95)	38 (95)	38 (95)
o White Irish	1 (1)	0 (0)	1 (3)
o Other white background	1 (1)	1 (3)	0 (0)
o Black Caribbean	2 (3)	1 (3)	1 (3)
BMI (kg/m^2^):			
o BMI= ≥ 30	22 (28)	12 (30)	10 (25)
o BMI = 25–29.9	29 (36)	13 (33)	16 (40)
o BMI = <25	29 (36)	15 (38)	14 (36)
Family history of breast cancer:			
o Yes	15 (19)	8 (20)	7 (18)
o No	65 (81)	32 (80)	33 (82)
Smoking:			
o Ever	33 (41)	12 (30)	21 (52)
o Never	47 (59)	28 (70)	19 (48)
Alcohol drinkers:	57 (71)	28 (70)	29 (72)
Current or previous co-morbidities:			
o Diabetes	3 (4)	2 (5)	1 (3)
o Hypertension	12 (15)	4 (10)	8 (20)
o High cholesterol	6 (8)	3 (8)	3 (8)
o Heart disease	4 (5)	2 (5)	2 (5)
o Vascular disease	2 (3)	1 (3)	1 (3)
o Asthma/chronic bronchitis	9 (11)	3 (8)	6 (15)
o Osteoarthritis	13 (16)	4 (10)	9 (23)
o Rheumatoid arthritis	3 (4)	2 (5)	1 (3)
o Kidney disease	2 (3)	0 (0)	2 (5)
Parity	69 (86)	36 (45)	33 (41)
Breast fed children	45 (56)	23 (58)	22 (55)
Currently menstruating	16 (20)	8 (23)	8 (20)
Oral Contraceptive (OC) use (current/previous)	64 (80)	30 (75)	34 (85)
Mean ± *s* years OC taken	9.2 ± 7.8	10.0 ± 7.9	8.5 ± 7.7
Previous/current use of HRT	21 (26)	9 (22)	12 (30)
Mean ± *s* years taking HRT	6.9 ± 4.9	5.9 ± 3.8	7.6 ± 5.5
Marital status:			
o Married/in relationship	65 (81)	36 (91)	29 (73)
o Single/divorced/separated/widowed	15 (19)	4 (9)	11 (27)
Highest qualification:			
o College degree/diploma and above	30 (40)	15 (38)	10 (27)
Employment status:			
o Employed full-time/part-time	41 (53)	21 (53)	21 (53)
IPAQ physical activity category:			
o Low activity	15 (19)	8 (20)	7 (18)
o Moderate activity	55 (69)	30 (75)	25 (63)
o High activity	10 (13)	2 (5)	8 (20)

Key: *HRT* Hormone Replacement Therapy

**Table 2:** Effect of physical activity (PA) intervention on PA and anthropometric variables (all PA data reported as MET-min∙wk^−1^)

			Within-group change at follow−up	Adjusted between-group change at follow−up		
	Baseline mean (SD)	Follow-up mean (SD)	Mean change (95 % CI)	Mean change (95 % CI)	ES	*p*-value
Total PA						
Intervention	1354.74 (1073.44)	1899.01 (985.84)	530.11 (203.35 to 856.86)	578.47 (76.09 to 1080.84)	.44	.024
Usual care	1974.60 (1478.57)	1968.19 (1133.87)	−49.66 (−532.95 to 433.62)	Reference		
Work-based PA						
Intervention	29.12 (117.59)	52.54 (145.10)	21.06 (−20.97 to 63.09)	−45.85 (−128.47 to 36.78)	−.10	.273
Usual care	203.85 (643.40)	241.24 (635.99)	66.91 (−17.76 to 151.58)	Reference		
Active transport PA						
Intervention	167.89 (160.67)	222.08 (181.90)	42.36 (−35.42 to 120.15)	23.14 (−88.82 to 135.10)	.10	.683
Usual care	223.56 (268.35)	255.16 (253.96)	19.20 (−83.73 to 122.13)	Reference		
Domestic PA						
Intervention	623.60 (627.00)	729.54 (663.90)	93.08 (−177.84 to 364.00)	153.61 (−219.72 to 526.93)	.23	.417
Usual care	850.68 (698.20)	793.10 (689.33)	−59.33 (−393.63 to 274.97)	Reference		
Leisure PA						
Intervention	478.76 (591.57)	875.42 (789.59)	414.03 (242.22 to 585.84)	382.18 (93.75 to 670.61)	.61	.010
Usual care	565.79 (671.65)	652.37 (529.02)	31.57 (−237.19 to 300.32)	Reference		
Walking PA						
Intervention	439.64 (416.43)	706.56 (789.59)	289.24 (105.74 to 472.74)	172.93 (−61.75 to 407.61)	.39	.147
Usual care	567.16 (472.40)	688.77 (528.71)	116.30 (−59.49 to 289.09)	Reference		
Moderate PA						
Intervention	695.10 (673.94)	856.24 (675.64)	142.49 (−126.52 to 411.49)	112.44 (−307.39 to 532.27)	.13	.597
Usual care	1087.60 (1020.28)	1126.04 (911.75)	30.61 (−376.54 to 437.77)	Reference		
Vigorous PA						
Intervention	142.03 (387.19)	275.65 (572.14)	122.11 (17.10 to 227.11)	264.07 (73.51 to 454.64)	.59	.007
Usual care	60.60 (143.22)	60.61 (143.22)	−143.06 (−340.84 to 54.72)	Reference		
Mass (kg)						
Intervention	70.86 (11.83)	69.43 (12.46)	−1.61 (−2.80 to−.42)	−1.62 (−3.16 to−.07)	−.14	.040
Usual care	69.15 (11.20)	69.19 (12.36)	−.00 (−1.03 to 1.04)	Reference		
BMI (kg/m^2^)						
Intervention	27.25 (4.69)	26.58 (4.93)	−.62 (−1.08 to −.17)	−.62 (−1.17 to −.06)	−.14	.030
Usual care	26.67 (4.04)	26.79 (4.2)	−.01 (−.41 to .40)	Reference		
Body fat %						
Intervention	35.88 (6.46)	36.24 (6.61)	.41 (−.55 to 1.37)	.34 (−.93 to 1.62)	.06	.594
Usual care	35.26 (5.90)	35.52 (6.26)	.05 (−.85 to .95)	Reference		

Key: SD indicates standard deviation; 95 % CI, 95 % confidence interval; ES, effect size (Cohen’s d; effect estimate/pooled baseline SD)

Baseline means (SD) are based on 80 participants (intervention = 40; usual care = 40); post-interventions and within-group change at follow-up means (SD) are based on 70 participants (intervention = 37; control = 33)

Except for the anthropometric measures, positive ES indicate effects in favour of the exercise intervention group

Between-group effects were assessed using linear mixed model analysis, adjusted for the value of the outcome variable at baseline

**Table 3:** Effect of PA intervention on HRQoL FACT-B and blood biomarker variables

			Within-group change at follow−up	Adjusted between-group change at follow−up		
	Baseline mean (SD)	Follow-up mean (SD)	Mean change (95 % CI)	Mean change (95 % CI)	ES	*p*-value
FACT-B						
Intervention	108.56 (21.97)	114.41 (21.48)	5.91 (1.88 to 9.93)	5.05 (.69 to 9.40)	.25	.024
Usual care	114.25 (18.97)	115.34 (17.57)	.56 (−3.43 to 4.56)	Reference		
FACT-G						
Intervention	85.75 (17.35)	88.03 (18.53)	2.62 (−2.72 to 7.96)	2.17 (−1.43 to 5.78)	.14	.234
Usual care	89.30 (13.23)	89.59 (16.84)	−.09 (−5.65 to 5.46)	Reference		
TOI						
Intervention	65.29 (15.09)	72.59 (15.13)	7.20 (4.47 to 9.93)	5.64 (2.33 to 8.95)	.39	.001
Usual care	71.13 (13.07)	73.25 (16.52)	2.13 (−1.89 to 6.14)	Reference		
PWB						
Intervention	22.03 (5.25)	25.54 (9.32)	3.43 (.58 to 6.29)	.63 (−.87 to 2.13)	.13	.404
Usual care	23.03 (4.39)	25.84 (9.18)	2.84 (−.15 to 5.84)	Reference		
SWB						
Intervention	24.35 (4.44)	23.70 (5.03)	−.54 (−1.40 to .32)	−.73 (−2.03 to .59)	.17	.276
Usual care	23.40 (4.19)	24.13 (4.13)	.19 (−1.00 to 1.37)	Reference		
EWB						
Intervention	18.93 (4.61)	20.11 (4.14)	1.24 (.46 to 2.03)	.20 (−.85 to 1.26)	.05	.701
Usual care	19.73 (3.74)	20.72 (3.30)	1.00 (.20 to 1.80)	Reference		
FWB						
Intervention	20.45 (6.10)	21.95 (4.41)	1.76 (.21 to 3.30)	1.90 (.24 to 3.55)	.36	.025
Usual care	23.15 (3.94)	22.88 (4.70)	−.16 (−1.25 to .94)	Reference		
BCS						
Intervention	22.81 (6.67)	25.24 (7.13)	2.15 (.98 to 3.32)	2.84 (.79 to 4.89)	.42	.007
Usual care	24.95 (6.79)	24.34 (6.21)	−75 (−2.81 to 1.31)	Reference		
TC (mmol∙L^−1^)						
Intervention	5.75 (1.30)	5.4 (1.09)	−.23 (−.49 to .04)	−.45 (−.71 to −.18)	−.38	.001
Usual care	5.79 (1.04)	5.93 (.91)	.22 (.05 to .38)	Reference		
HDL (mmol∙L^−1^)						
Intervention	1.65 (.30)	1.62 (.33)	−.02 (−.12 to 0.79)	−.06 (−.15 to .04)	−.19	.264
Usual care	1.59 (.34)	1.60 (.30)	.04 (−.03 to .10)	Reference		
LDL (mmol∙L^−1^)						
Intervention	3.44 (1.15)	3.18 (1.01)	−.19 (−.42 to .04)	−.30 (−.56 to −.04)	−.30	.023
Usual care	3.56 (.84)	3.64 (.84)	.11 (−.11 to .32)	Reference		
TC/HDL-C ratio (mmol∙L^−1^)						
Intervention	3.61 (1.12)	3.47 (.93)	−.09 (−.36 to .09)	−.13 (−.40 to .14)	−.12	.337
Usual care	3.79 (1.00)	3.83 (.90)	.04 (−.19 to .26)	Reference		
Trig (mmol∙L^−1^)						
Intervention	1.43 (.75)	1.31 (.58)	−.08 (−.21 to .05)	−.10 (−.27 to .07)	−.13	.240
Usual care	1.52 (.85)	1.52 (.73)	.02 (−.14 to .18)	Reference		
Glucose (mmol∙L^−1^)						
Intervention	4.94 (.85)	4.81 (.52)	−.14 (−.36 to .09)	−.07 (−.38 to .25)	−.05	.683
Usual care	5.27 (1.96)	5.32 (2.20)	−.08 (−.40 to .25)	Reference		
Insulin (pmol∙L^−1^)						
Intervention	38.37 (34.61)	37.40 (28.64)	−1.03 (15.37 to 13.31)	8.31 (−12.31 to 28.95)	.20	.425
Usual care	45.45 (48.69)	37.34 (40.60)	−9.84 (−29.76 to 10.08)	Reference		
HOMA						
Intervention	1.60 (1.18)	1.78 (.88)	.07 (−.62 to .76)	.42 (−.88 to 1.73)	.27	.520
Usual care	2.18 (1.83)	1.90 (2.09)	−.41 (−2.09 to 1.26)	Reference		

Key: FACT-G = PWB + SWB + EWB + FWB; FACT-B = FACT-G + BCS; TOI = PWB + FWB + BCS

Baseline means (SD) are based on 80 participants except for HOMA (*N* = 52; intervention = 27; control = 25); Post-interventions and with-group change at follow-up means (SD) are based on 70 participants (intervention = 37; control = 33), except HOMA (*N* = 38; Intervention = 20; control = 18)

Except for the blood measures (Higher scores represent better quality of life), positive ES indicate effects in favour of the exercise intervention group

Between-group effects were assessed using linear mixed model analysis including the measurements obtained at baseline and post-intervention, adjusted for the value of the outcome variable at baseline

### PA outcomes

When adjusted for baseline levels, the intervention resulted in a significant but small increase in total PA compared to the usual care group (*p* < .05; *d* = .44) (Table 2). In particular, leisure PA and vigorous PA increased significantly and moderately in the intervention compared with the usual care group over the intervention period (both *p* ≤ .01; *d* ≤ .60). The per-protocol, magnitude-based inference (adjusted for baseline levels) analysis revealed the effect of the PA intervention was *likely* to have been beneficial (80 % likelihood of a beneficial effect) on moderate PA despite a non-significant main effect, compared with the usual care (Table 4). However, the effect of the intervention was possibly beneficial on all other PA (50 % likelihood of a beneficial effect), except for a possible negative effect on work-based and active transport.

**Table 4:** Changes in performance and anthropometric measures in experimental and control groups and qualitative inferences about the intervention effects

Variable	Change in measure (%) from baseline to post-intervention				
	Intervention mean (SD)	Usual care mean (SD as a CV)	Between group difference (90 % CI)	Effect size (*d*)	Qualitative inference (% likelihood of at least a small effect)
Total PA	55.9 (209.5)	17.3 (93.0)	32.9 (−9.0 to 94.0)	.31 (−.10 to .72)	Possibly beneficial (67)
Work-based PA	−6.3 (814.8)	51.2 (327.1)	−56.2 (−84.0 to 19.8)	−.33 (−.73 to .07)	Possibly decreases (52)
Active transport PA	−24.6 (783.9)	72.3 (1452.7)	−44.7 (−79.9 to 52.2)	−.23 (−.63 to .16)	Possibly decreases (70)
Domestic PA	81.3 (652.3)	−11.4 (768.2)	104.6 (−12.5 to 378.7)	.37 (−.07 to .81)	Possibly beneficial (74)
Leisure PA	408.0 (1208.6)	208.9 (1615.0)	64.8 (−44.0 to 384.9)	.19 (−.23 to .61)	Possibly beneficial (50)
Walking PA	76.2 (851.2)	70.7 (916.4)	3.3 (−59.0 to 160.1)	.02 (−.47 to .50)	Possibly beneficial (51)
Moderate PA	71.1 (477.9)	−18.2 (527.5)	109.1 (−.2 to 338.2)	.41 (.00 to .83)	Likely beneficial (80)
Vigorous PA	137.6 (2078.0)	33.6 (868.1)	77.8 (−39.2 to 420.0)	.22 (−0.19 to .62)	Possibly beneficial (53)
Mass	−2.3 (4.7)	−.1 (4.1)	−2.2 (−3.9 to −.5)	−.13 (−.24 to −.03)	Unlikely beneficial (14)
BMI	−2.3 (4.6)	−.1 (4.1)	−2.2 (−3.9 to −.5)	−.14 (−.25 to −.03)	Unlikely beneficial (18)
Body fat %	1.3 (8.0)	−.1 (7.5)	1.4 (−1.6 to 4.4)	.08 (−.09 to .25)	Unlikely increases (11)

Key: *CV *= coefficient of variation

Beneficial effect reflects an increase in PA measures and a decrease in anthropometric measures

Regarding categorical PA data, 88 % (*n* = 7/8) and 12 % (*n* = 1/8) of the participants in the intervention group categorised as low activity at baseline, moved to the moderate and high activity category post-intervention, respectively. In the usual care group, 50 % (*n* = 2/4) remained in the low activity category while only one participants each moved from low to moderate and high activity categories, post-intervention.

### Anthropometric outcomes

The intervention group experienced trivial but significant decreases in both body mass and BMI from baseline to post-intervention compared with the usual care group (both *p* < .05, *d* < .02). However, no significant change in body fat % was observed (Table 2).

### HRQoL outcomes

Analyses highlighted a significant but small improvement in FACT-B, TOI, FWB and BCS scores in the PA group compared with the usual care group over the 6-month intervention period (*p* < .05 and *d* < .50, respectively). No significant differences between PA and usual care groups were found for any of the other HRQoL variables (Table 3). Magnitude-based inference adjusted analysis of study completers revealed the effect of the PA intervention was only *possibly* to have been beneficial (80 % likelihood of a beneficial effect) on all HRQoL, compared with the usual care (Table 5).

**Table 5:** Changes in HRQoL and blood biomarkers measures in experimental and control groups and qualitative inferences about the intervention effects

Variable	Change in measure (%) from baseline to post-intervention				
	Intervention mean (SD)	Usual care mean (SD as a CV)	Between group difference (90 % CI)	Effect size (*d*)	Qualitative inference (% likelihood of at least a small effect)
Fact-B	5.9 (10.8)	2.1 (7.9)	3.7 (.0 to 7.5)	.18 (.00 to .35)	Possibly beneficial (59)
Fact-G	16.2 (85.1)	2.7 (8.8)	13.1 (−4.9 to 34.6)	.34 (−.14 to .82)	Possibly beneficial (69)
TOI	4.8 (31.1)	1.6 (10.2)	3.1 (−4.8 to 11.8)	.13 (−.21 to .47)	Possibly beneficial (36)
BCS	8.8 (18.5)	1.0 (28.1)	7.7 (−1.2 to 17.5)	.22 (−.04 to .47)	Possibly beneficial (54)
PWB	9.2 (16.2)	7.6 (14.6)	1.5 (−4.2 to 7.5)	.07 (−.19 to .33)	Unlikely beneficial (20)
SWB	−2.5 (12.3)	.7 (13.3)	−3.2 (−7.8 to 1.6)	−.15 (−.37 to .07)	Possibly decreases (36)
EWB	5.6 (13.5)	5.6 (9.7)	−.0 (−4.3 to 4.5)	.00 (−0.19 to .19)	Very unlikely beneficial (5)
FWB	6.2 (20.4)	−1.3 (15.0)	7.6 (.6 to 15.2)	.26 (.02 to .50)	Possibly beneficial (66)
TC	−3.5 (10.5)	3.2 (6.7)	−6.5 (−9.6 to −3.3)	−.41 (−.62 to −.21)	Very likely beneficial (95)
HDL-C	−.7 (11.0)	1.0 (6.7)	−1.7 (−5.0 to 1.9)	−.14 (−.42 to .15)	Possibly beneficial (35)
LDL-C	−4.5 (14.9)	2.5 (12.8)	−6.8 (−11.6 to −1.8)	−.31 (−.55 to −.08)	Likely beneficial (79)
TC/LDL-C ratio	−2.3 (14.5)	1.6 (11.3)	−3.8 (−8.5 to 1.0)	−.19 (−.43 to .05)	Possibly beneficial (47)
Trig	−3.5 (16.3)	1.8 (16.4)	−5.2 (−10.9 to .8)	−.20 (−.42 to .03)	Possibly beneficial (49)
Glucose	−2.9 (6.7)	−6.1 (40.6)	3.4 (−6.7 to 14.5)	.14 (−.30 to .59)	Possibly beneficial (42)
Insulin	−3.6 (87.3)	−24.2 (145.4)	27.2 (−7.1 to 74.3)	.31 (−.09 to .70)	Possibly increases (67)
HOMA	−4.5 (39.5)	0.7 (61.6)	−5.2 (−26.6 to 22.5)	−.12 (−.72 to .47)	Possibly beneficial (41)

Key: *CV* = coefficient of variation

Beneficial effect reflects an increase in HRQoL measures and a decrease in blood biomarkers

Chi-square analysis of the FACT-B, FACT-G, TOI, and BCS variables revealed significant associations between intervention and usual care groups and the number of participants who experienced minimum clinically important increases in TOI, *χ*^2^ (1) = 8.34, *p* = .004, and BCS, *χ*^2^ (1) = 6.19, *p* = .013. More than twice as many participants in the intervention group experienced minimum clinically important improvements in BSC and TOI between baseline and post-intervention compared with the usual care group (57 %, *n* = 21/37 vs. 27 %, *n* = 9/33; and 65 %, *n* = 24/37 vs. 30 %, *n* = 10/33). No significant associations were found between intervention and usual care groups and the number of participants who experienced minimum clinically important changes in FACT-B, *χ*^2^ (1) = 1.67, *p* = .23, and FACT-G, *χ*^2^ (1) = 0.31, *p* = .63.

### Blood biomarker outcomes

We found significant but small reductions in TC and LDL-C concentrations in the PA group compared with the usual care group over the 6-month intervention period (*p* < .05 and *p* < .01, respectively, and *d* < .05) but not for any of the other parameters studied (Table 3). Magnitude-based inference adjusted analysis revealed the effect of the PA intervention was *likely* and *very likely* to have been beneficial (>75 % likelihood of a beneficial effect) on TC and LDL-C, respectively, compared with the usual care (Table 5).

## Discussion

Breast cancer survivors who received a home-based PA intervention significantly increased our primary outcome, self-reported total PA compared with usual care. We also found further significant improvements in leisure and vigorous PA, body mass, BMI, HRQoL (FACT-B, TOI, FWB, and BCS) and TC and LDL-C concentrations in the intervention compared with usual care. All of the significant improvements above were found to have small effect sizes, apart from the moderate effects observed for leisure and vigorous PA. However, the difference in improvement in total PA for the intervention group (578 MET-min∙wk^−1^) compared to the usual care group was close to the recommended PA guidelines of 600 MET-min∙wk^−1^, i.e. 5 × 30 min of moderate PA). Therefore, this improvement would result in more breast cancer survivors meeting recommended PA guidelines, and possibly deriving associated benefits of reduced risk of mortality and recurrence [9–12]. Of note, more participants in the intervention group experienced minimum clinically important improvements in TOI and BCS compared with the usual care group. However, we observed no significant improvements in any other PA variables, body fat, and other HRQoL and blood biomarker variables.

Our findings of increases in total, leisure-based, and vigorous PA are consistent with previous US home-based PA interventions with an additional PA counselling element [17, 20, 22]. All of these trials were relatively short in duration (12 weeks) compared with the duration of the current study (6 months). The increases in PA found in the current study were encouraging given the larger sample size of invasive breast cancer survivors. However, unlike two previous studies [20, 27], we found no significant differences in self-reported walking from baseline to post-intervention in the intervention group compared with the usual care group. This was possibly due to contamination in the usual care group since these individuals were made aware of recommended PA guidelines at baseline, as it was thought unethical to withhold this information considering the potential health benefits associated with PA. Therefore, being part of the current study may have increased the awareness of health benefits associated with PA in the usual care group and resulted in increased walking activity. Another possible reason for this is that the IPAQ assesses walking in occupational and active transport domains as well as leisure domains, in which usual care participants engaged in more than the intervention participants. Similarly, a greater amount of occupational and active transport may also explain the non-significant between-group differences in moderate PA, although the per-protocol analysis revealed a *likely beneficial* effect of the intervention on moderate PA. It is also important to note that, on average, the PA levels of the intervention group were lower than that of the usual care group at baseline, and therefore, it can be argued that they had a greater room for improvement. However, the higher self-reported PA levels of the usual care group was largely the result of three participants in this group who reported much higher PA levels (≥5000 MET-min∙wk^−1^) compared to other participants. Therefore, with the exception of these three participants the levels of PA were similar in both groups, as evidenced by the number of participants in the low and moderate PA categories in each group (see Table 1).

Unlike similar previous studies, we found significant reductions in body mass and BMI [17, 20, 22]. Although the effects of the intervention compared with usual care could be considered trivial for both outcomes, it does represent at the least, more effective weight management. The significant albeit small reductions in mass and BMI were surprising given that the intervention did not focus on weight loss and did not involve any calorie restriction. However, previous research has found positive associations between PA and healthy eating behaviours [44], which in turn may have had a beneficial effect on body mass and BMI. In addition, this finding could be due in part to the longer duration of the current study compared with the earlier studies (6 months vs. 12 weeks) [17, 20, 22, 27]. However, we found no significant improvements in body fat % despite the improvements in mass and BMI. It is possible that the method of assessing body fat %, bioelectrical impedance is not a precise enough method to measure small changes in body fat over time [45].

We observed significant small increases in the HRQoL variables, FACT-B, TOI, FWB and BCS in the intervention group compared to the usual care group. In addition, a greater proportion of participants in the intervention group achieving minimum clinical significant improvements in BSC and TOI, which indicates that our intervention may have specific benefits for breast cancer survivors given that higher BCS scores indicate fewer breast cancer-specific symptoms, such as ‘shortness of breath’, ‘change in weight’ and ‘effect of stress on illness’, and higher TOI scores indicate both greater physical and functional well-being and fewer breast cancer-specific symptoms. A methodologically similar study reported significantly greater improvements for social well-being in the intervention group versus usual care group, but no significant improvements were found in the other HRQoL variables [17]. Significant improvements in the FACT-B variable in the intervention group versus usual care group was reported by an earlier home-based PA trial involving breast cancer survivors, which did not have a counselling component [26]. The reasons for the differences between previous studies are unclear. However, it is likely that the breast cancer stage, treatment received and both the time since diagnosis and the end of treatment may influence participant’s responses to the items with the FACT questionnaire.

Our findings of significant but small reductions in TC and LDL-C were encouraging given that the existing literature investigating the prevention of cardiovascular disease (CVD) emphasizes the role of TC and LDL-C with a supplementary role for HDL-C and a modest role for TG [46–48]. Evidence supports our finding that increased PA can favourably influence lipid profiles [49–51]. The effect of aerobic exercise on glucose-insulin dynamics is unclear due to a lack of agreement between available studies [52–55]. We may not have found reductions in glucose, insulin, and IR because of an insufficient sample size to detect differences between groups as the trial was not powered to detect changes in these outcomes, an insufficient reduction in body fat [55], and/or the fact that the majority of participants did not have diabetes [56].

The strengths of the current study include its randomised design, the independent randomisation, a pragmatic intervention and the intention-to-treat approach. We also recruited participants over two full calendar years; therefore, it is unlikely that our results were influenced by the seasonal changes in PA suspected in previous research [26]. The limitations of this study include lack of controlling for increased risk of type I errors when making multiple comparisons. Moreover, self-report measures, such as IPAQ, require participants to recall past activity, are a subjective means of estimating individual PA levels and are reliant on the individuals’ ability to remember levels of exposure [57]. Outcomes were assessed by a fully trained exercise scientist, who followed an objective, standardized assessment protocol. However, the scientist was not blinded to group allocation which may have introduced measurement bias. In addition, there was evidence of some contamination in the usual care group. Six of the usual care group increased their PA levels enough to move to a higher PA category from baseline to post-intervention. This contamination may have been because we informed participants in the usual care of the current recommended PA guidelines and we did not discourage them from engaging in PA. We did not control for possible changes in the dietary habits of participants, and it is possible that participants in the intervention group may have also changed to healthier eating behaviours when becoming more physically activity.

## Conclusions

Within the context of these limitations, we found that a home-based PA intervention resulted in significant but small to moderate favourable effects on self-reported PA, body mass, BMI, HRQoL, TC and LDL-C. The results of the trial were promising given that the intervention was relatively brief, pragmatic and highly feasible given that it was home-based and consisted of a single in-person counselling session followed by three support telephone calls. The portability and feasibility of the current intervention means it could be implemented within the NHS framework of breast cancer treatment and follow-up both in the primary and secondary care settings. This has the potential to capture the maximum number of breast cancer survivors can benefit with minimal burden to staff.

## Availability of data and materials

The datasets supporting the conclusions of this article are available in the Figshare repository (https://figshare.com/articles/Randomised_controlled_trial_of_a_home_based_physical_activity_intervention_in_breast_cancer_survivors/3082987).

## Abbreviations

BCS: Breast cancer subscale score
BMI: Body mass index
EWB: Emotional well-being
FACT-B: FACT-breast
FACT-G: Functional assessment of cancer therapy - general
FWB: Functional well-being
HDL-C: High-density lipoprotein
HOMA: Homeostasis Model Assessment
HRQoL: Health-related quality of life
HRT: Hormone Replacement Therapy
IR: Insulin resistance
LDL-C: Low-density lipoprotein cholesterol
PA: Physical activity
PWB: Physical well-being
RCT: Randomised controlled trials
SWB: Social well-being
TC: Total cholesterol
TG: Triglycerides
TOI: Trial outcome index
